# Cirsilineol Inhibits the Proliferation of Human Prostate Cancer Cells by Inducing Reactive Oxygen Species (ROS)-Mediated Apoptosis

**DOI:** 10.1155/2022/7975664

**Published:** 2022-07-09

**Authors:** Shadma Wahab, Abdulrhman Alsayari, Abdullatif Bin Muhsinah, Irfan Ahmad, Md. Sarfaraj Hussain, Jewel Mallick

**Affiliations:** ^1^Department of Pharmacognosy, College of Pharmacy, King Khalid University, Abha 61421, Saudi Arabia; ^2^Complementary and Alternative Medicine Unit, College of Pharmacy, King Khalid University, Abha 6142, Saudi Arabia; ^3^Department of Clinical Laboratory Sciences, College of Applied Medical Sciences, King Khalid University, Abha 61421, Saudi Arabia; ^4^Lord Buddha Koshi Pharmacy College of Pharmacy, Baijanathpur NH 107, Saharsa 852201, Bihar, India; ^5^Department of Pharmacy, BGC Trust University Bangladesh, Chittagong 4381, Bangladesh

## Abstract

Cirsilineol has been reported to exhibit anticancer effects against several human cancer cell lines. The present study was designed to evaluate the anticancer effects of cirsilineol against the human DU-145 prostate cancer cells. The results showed that cirsilineol suppressed the proliferation of DU-145 cancer cells in a dose-dependent manner with minimal cytotoxic effects against the normal cells. The IC_50_ of cirsilineol was found to be 7 *μ*M and 110 *μ*M against prostate cancer DU-145 and normal HPrEC prostate cells, respectively. Acridine orange and ethidium bromide (AO/EB) staining showed that cirsilineol induced apoptosis in DU-145 prostate cancer cells. The Annexin V/PI staining further confirmed the induction of apoptosis in DU-145 cells. The western blot analysis showed that cirsilineol suppressed the expression of Bax and upregulated the expression of Bcl-2 in prostate cancer DU-145 cells. Moreover, cirsilineol caused a dose-dependent increase in reactive oxygen species (ROS) levels in prostate cancer. Wound healing and Transwell assays showed that cirsilineol inhibits migration and invasion of DU-145 prostate cancer cells. Summing up, the results suggest that cirsilineol suppresses the proliferation of prostate cancer cells and may prove to be a beneficial lead molecule for the development of chemotherapy for prostate cancer.

## 1. Introduction

The growing incidence of human cancers and the associated mortalities has compelled the search for novel drugs that suppress the proliferation of cancer cells while having negative effects on normal cells [1]. Many of the previous anticancer agents have been reported to exhibit toxic effects not only against the cancer cells but also against the normal cells [2]. Currently, a lot of research is being conducted to identify anticancer agents from plants. Plants have been utilized for the management of several human diseases since times immemorial. As a part of folklore, several plants or plant products have been used for health-promoting effects [3]. In 2017, around 1.7 million new cancer cases and 0.6 million cancer-related deaths were reported [4]. Recently, numerous molecules derived from plants have been evaluated against human cancer cells and experimental animals. This has resulted in a dynamic increase in the number of newly discovered natural compounds. In 2006, about 50,000 such molecules were known, whereas, in 2014, the number of newly discovered molecules increased to approximately 326,000 [5, 6]. Cirsilineol is a trimethoxy and dihydroxy flavones type of flavonoid that has been previously isolated from several plant species such as *Artemisia vestita* [7, 8]. Several studies have reported the antioxidant, antiinflammatory, and anticancer potential of cirsilineol [8]. In a recent study, it was found to halt the proliferation of squamous lung carcinoma cells via the promotion of apoptosis [9]. Additionally, cirsilineol has been found to exhibit gastroprotective effects against the hydrochloric acid/ethanol-induced ulceration in rat models *in vivo* [10]. With this background, the present study was designed to evaluate the anticancer effects of cirsilineol against the human DU-145 prostate cancer cells and unveil the underlying molecular mechanism. Herein, we report that cirsilineol suppresses the growth of prostate cancer cells via the induction of ROS-mediated apoptosis. This study will form the basis for the establishment of cirsilineol as a lead molecule for the development of prostate cancer chemotherapy.

## 2. Materials and Methods

### 2.1. Cell Lines and Culture Conditions

The human DU-145 prostate cancer cells were purchased from the American Type Culture Collection (ATCC, USA). Both the cell lines were propagated using RPMI-1640 (Gibco, Carlsbad, CA, USA) containing 10% fetal bovine serum (FBS, Gibco, Carlsbad, CA, USA) and 1% penicillin/streptomycin (WelGENE).

### 2.2. Cell Viability Assessment

After their incubation with varying cirsilineol concentrations (0 to 100 *μ*M) for 24 h at 37° in 96-well plates, DU-145 cancer cells and HPrEC normal cells were added with 15 *μ*L (3 -(4, 5-dimethylthiazol-2-yl)-2,5-diphenyltetrazolium bromide) (MTT) reagent (Sigma-Aldrich) and their reincubation was performed at 37°C for 4 h. After harvesting, dimethyl sulfoxide (DMSO) was used for resuspending the cell pellets. In the end, the OD_570_ value was recorded for each sample using a spectrophotometer.

### 2.3. Colony Formation Assay

For the clonogenic assay, 5000 DU-145 cancer cells without or with cirsilineol treatment (3.5 *μ*M, 7 *μ*M, or 14 *μ*M) suspended in 1 mL Dulbecco's Modified Eagle Medium (DMEM) were plated in each well of a 6-well plate. The cells were grown for 2 weeks at 37°C with 5% CO_2_. After removing the culture medium, the clones were treated with ethanol and subsequently stained using 0.1% crystal violet and then photographed.

### 2.4. Acridine Orange (AO) and Ethidium Bromide (EB) Staining

DU-145 prostate cancer cells were seeded into a 96-well plate with a cellular density of 5 × 10^5^ cells/well. The cells were incubated with different concentrations of cirsilineol (0 *μ*M, 3.5 *μ*M, 7 *μ*M, or 14 *μ*M) for 24 h at 37°C. Afterward, the cells were collected through centrifugation, washed with phosphate-buffered saline (PBS), and fixed using 70% ethanol for 1 h at room temperature. The cells were then again PBS washed and administered with 0.2% Triton X−100. The cancer cells were then stained with a solution of AO/EB reagent (Solarbio Biotechnology, China) for 20 min at room temperature. Finally, cells were given PBS wash and then examined under a fluorescent microscope.

### 2.5. Annexin V/PI Staining Assay

The Annexin V-FITC/PI staining method was used to more precisely study the apoptosis of cirsilineol-treated (0 *μ*M, 3.5 *μ*M, 7 *μ*M, or 14 *μ*M) DU-145 cancer cells. Following their administration with varied cirsilineol treatments for 24 h, the cancer cells were harvested and washed with PBS twice. Afterward, the cells were stained with Annexin V-FITC (Thermo Fisher Scientific, Waltham, MA) and propidium iodide (Thermo Fisher Scientific, Waltham, MA) solutions. Finally, the apoptosis of DU-145 cancer cells was studied with the help of FACSCanto II (BD Biosciences, San Jose, CA) flow cytometer system.

### 2.6. Reactive Oxygen Species (ROS) and Mitochondrial Membrane Potential (MMP) Determination

DU-15 cells at the density of 2 × 10^5^ cells/well were seeded in a 6-well plate and allowed to incubate at 37°C for 24 h. Subsequently, the cells were treated with 0, 3.5, 7, or 14 *μ*M cirsilineol at 37°C. Then, the cells were PBS washed and treated with 500 *μ*L of 2′-7′-dichlorofluorescin diacetate (DCFH-DA) (10 *μ*M) for ROS estimation and (3,3′-dihexyloxacarbocyanine iodide) (DiOC6) (1 *μ*mol/L) for MMP at 37°C in a dark room for 30 min. The final determination of ROS and MMP was performed by flow cytometry.

### 2.7. Wound-Healing Assay

The DU-145 cancer cells without or with cirsilineol (7 *μ*M) were cultured in the wells of a 6-well plate till 80% confluence. The cell surface was then wounded with a 200 *μ*l pipette tip and photographed. The 6-well plate was incubated for 24 h at 37°C. Using a microscope, the wound was again photographed.

### 2.8. Transwell Invasion Assay

The invasion of DU-145 cancer cells without or with cirsilineol (7 *μ*M) was estimated by performing the Transwell assay, wherein the relative number of cancer cells crossing a porous polycarbonate membrane of the BioCoat Matrigel invasion chamber (BD Bioscience), under chemo-attraction of higher serum concentration, was analyzed. Here, 5 × 10^4^ cancer cells were plated into the upper chamber while DMEM with 10% FBS was added into the lower chamber. The incubation of 24 h at 37°C was then given. The cells which had traversed the polycarbonate membrane were fixed with methanol, stained with crystal violet, and examined with a microscope.

### 2.9. Western Blotting

The DU-145 cancer cells without or with cirsilineol treatment (3.5 *μ*M, 7 *μ*M, or 14 *μ*M) were digested with RIPA lysis buffer (Sigma-Aldrich, Germany) for total protein isolation. The proteins after quantification were resolved on 10% SDS‐polyacrylamide gels which were blotted to nitrocellulose membranes. Exposure to specific primary antibodies Bax (sc-7480, Santa Cruz, CA, USA), Bcl-2 (sc-23960, Santa Cruz, CA, USA), and Actin (sc-58673, Santa Cruz, CA, USA) was given to the membranes in dark at 4°C overnight. This was followed by their treatment with horseradish peroxidase-conjugated secondary antibodies at room temperature for 2 h. Specific protein bands were then detected by using FluroChem E-System (Protein Simple, Silicon Valley). *β*-Actin was used as an internal control.

### 2.10. Statistical Analysis

The experiments were performed in triplicate and expressed as mean ± SD. Student's *t*-test was used to carry out the statistical analysis. *P* < 0.05 was considered to be a measure of statistically significant difference.

## 3. Results

### 3.1. Cirsilineol Inhibited the Proliferation of DU-145 Prostate Cancer Cells

The prostate cancer cells (DU-145), as well as, normal HPrEC were incubated with variable treatment concentrations (0 to 100 *μ*M) of cirsilineol (Figure 1(a)) for 24 h at 37°C to analyze the effect of changing cirsilineol concentrations on the DU-145 and HPrEC cell proliferation. Cirsilineol administration though minimized the proliferation of DU-145 cancer, as well as the primary prostate epithelial cells (HPrEC), but the DU-145 cancer cells were shown to be affected more prominently as compared to the normal plasma cells (Figure 1(b)). The IC_50_ of cirsilineol was 7 *μ*M against DU-145 cancer cells. On the other hand, it was more than ∼16 times higher than the normal HPrEC cells (110 *μ*M) which signified the selective and potent growth inhibitory action of cirsilineol against the DU-145 prostate cancer cells.

### 3.2. Cirsilineol Inhibited the Colony Formation of DU-145 Prostate Cancer Cells

To further look into the growth declining action of cirsilineol against the prostate cancer cells, the DU-145 cancer cells were incubated at 37°C with (3.5 *μ*M, 7 *μ*M, or 14 *μ*M) or without cirsilineol and subjected to colony formation assay. The results showed that cirsilineol suppressed the colony formation of DU-145 cells in a dose-dependent manner (Figure 2(a)). The colony formation was inhibited by 73% at 14 *μ*M cirsilineol (Figure 2(b)).

### 3.3. Cirsilineol Treatment Induced Apoptosis in DU-15 Prostate Cancer Cells

To specifically figure out the underlying mechanism for the antiproliferative action of cirsilineol against the prostate cancer cells, the DU-145 prostate cancer cells were administered with 0 *μ*M, 3.5 *μ*M, 7 *μ*M, or 14 *μ*M for 24 h. Next, the cells were incubated with AO/EB dual staining mix, and notably, the relative percentage of prostate cancer cells stained with acridine orange (AO) was shown to be increasing with increased cirsilineol concentrations (Figure 3). Moreover, the Annexin V-FITC/PI staining combined with flow cytometry showed that the DU-145 prostate cancer cells were induced with apoptotic cell death by cirsilineol treatments (Figure 4(a)). The relative abundance of apoptotic prostate cancer cells was shown to be increasing with increasing concentrations of cirsilineol (0 *μ*M–18 *μ*M). The percentage of early and late apoptotic cells increased from 5% in untreated cells to 21.22% at a 14 *μ*M concentration of cirsilineol. Western blotting showed that the expression of Bax increased and that of Bcl-2 decreased in a dose-dependent manner (Figure 4(b)). Next, we also examined the ROS and MMP levels in cirsilineol-treated cells and it was found that cirsilineol caused a significant increase in ROS levels which was accompanied by loss of MMP (Figures 4(c) and 4(d)). These effects of cirsilineol on reactive oxygen species (ROS) and mitochondrial membrane potential (MMP) were concentration-dependent. Thus, these results suggest the proapoptotic activity of cirsilineol in prostate cancer.

### 3.4. Cirsilineol Suppressed the Migration and Invasion of DU-145 Prostate Cancer Cells

The effect of the *in vitro* administration of cirsilineol on the migration and invasion of the DU-145 prostate cancer cells was also assessed. The migration of untreated DU-145 cancer cells and those treated with 7 *μ*M cirsilineol was analyzed by wound-healing assay. It was found that cirsilineol suppressed the migration of the DU-145 cells (Figure 5). The wound-healing potential was significantly higher for untreated cells while it was invariably lower for the cirsilineol-treated cells. The effects of cirsilineol were also examined on the invasion of the DU-145 prostate cancer cells and it was found that the migration of prostate cancer cells decreased in a dose-dependent manner (Figure 6).

## 4. Discussion

Prostate cancer has a significant mortality across the globe and is becoming one of the common causes of cancer-related deaths [11]. In 2021, prostate cancer caused around 30,000 deaths out of the 248000 confirmed prostate cancer cases [12]. Although the 5-year survival for prostate cancer is around 99% at the initial stages, however, the diseases is generally incurable at advanced stages [13]. Therefore, there is a pressing need to identify efficient molecules from natural sources for the management of prostate cancer. Numerous studies centered at exploration of the medicinal value of natural compounds have proposed that these compounds might emerge as key players against several human diseases including the deadly cancers [14]. There is growing support for natural compounds to replace the synthetic chemical compounds for their relatively minimal undesirable effects on the normal body cells [15]. In a similar type of observation, cirsilineol was shown to significantly reduce the growth of prostate cancer cells *in vitro,* and on the one hand, it had little effect on the viability of the normal prostate cells. These findings are confirmation of several other studies, wherein cirsilineol has been reported to suppress the growth of several cancer cells. For example, Jing et al. showed that cirsilineol suppresses glioma cell growth via induction of apoptosis [16]. Similarly, Sheng et al. reported inhibition of the growth of different cancer cells by cirsilineol [17]. Apoptosis is an important mechanism by which defective or cancer cells are eliminated from the body [17]. Several anticancer agents have been reported to inhibit the growth of cancer cells by inducing apoptosis [18, 19]. For instance, cisplatin, a well-known anticancer drug, has been shown to induce apoptosis in cancer cells [20, 21]. In the present study, it was found that cisplatin-induced apoptosis in prostate cancer cells suggests the potential of cirsilineol in the management of prostate cancer. Bax and Bcl-2 are important biomarker proteins of apoptosis [22]; we examined the expression of these proteins in cirsilineol-treated prostate cancer cells and found that cirsilineol suppresses the expression of Bcl-2 and enhances the expression of Bax further confirming the induction of apoptosis in prostate cancer cells.

Cell migration and invasion are initial steps in the metastasis of cancer cells [23]. The drugs which can inhibit the metastasis of cancer cells are considered of utmost importance [24]. In the present study, we found that cirsilineol suppresses the migration and invasion of prostate cancer cells indicative of its antimetastatic potential. These findings are in agreement with previous investigations, wherein many flavonoids have been found to suppress the migration and invasion of cancer cells [25]. Taken together, these results suggest the potential of cirsilineol in the management of human prostate cancer. However, further studies are required to confirm these findings.

## 5. Conclusion

The findings of the present study revealed that cirsilineol suppresses the proliferation of prostate cancer cells via induction of apoptosis. Moreover, cirsilineol also suppressed the migration and invasion of prostate cancer cells. Collectively, the results indicate the potential of cirsilineol in the management of prostate cancer. However, more studies involving many cell lines and *in vivo* systems are urgently required.

## Figures and Tables

**Figure 1:** Cirsilineol inhibits proliferation of prostate cancer cells. (a) Chemical structure of cirsilineol. (b) MTT assay showing the effect of cirsilineol on the proliferation of the DU-145 and HPrEC cells. Experiments were performed in triplicate (^*∗*^*P* < 0.05).

**Figure 2:** Cirsilineol inhibits colony formation of prostate cancer cells. (a) Colony formation by the DU-145 cells at different concentrations of cirsilineol. (b) Percentage of colonies at each concentration of cirsilineol. Experiments were performed in triplicate (^*∗*^*P* < 0.05).

**Figure 3:** AO/EB staining of cirsilineol treated the DU-145 prostate cancer cells showing signs of apoptosis. Arrows depict apoptotic cells. Experiments were performed in triplicate.

**Figure 4:** Cirsilineol induces apoptosis in prostate cancer cells. (a) Annexin V/PI assay showing the percentage of apoptotic cells at indicated concentrations of cirsilineol. (b) Expression of Bax and Bcl-2 proteins at indicated concentrations of cirsilineol as determined by western blotting. (c) Cirsilineol increased ROS levels in DU-15 cells. (d) Cirsilineol decreased MMP levels in DU-15 cells. Experiments were performed in triplicate (^*∗*^*P* < 0.05).

**Figure 5:** Cirsilineol inhibits migration of prostate cancer cells. Wound healing assay showing migration of DU-145 cells treated with 0 or 12 *μ*M cirsilineol for 24 h. Experiments were performed in triplicate.

**Figure 6:** Cirsilineol inhibits the invasion of prostate cancer cells. Transwell assay showing invasion of DU-145 cells at indicated concentrations of cirsilineol. Experiments were performed in triplicate.

## Data Availability

All data used to support the findings of this study are included within the article.
